# Propofol Causes Consciousness Loss by Affecting GABA-A Receptor in the Nucleus Basalis of Rats

**DOI:** 10.1155/2020/9370891

**Published:** 2020-02-20

**Authors:** Yunlong Xing, Kai Li, Yuan Jiao, Zinan Li

**Affiliations:** ^1^Department of Plastic Surgery, China-Japan Union Hospital of Jilin University, Changchun 130033, China; ^2^Department of Anesthesiology, China-Japan Union Hospital of Jilin University, Changchun 130033, China

## Abstract

**Objective:**

Propofol is a classical anesthetic and induces consciousness loss, and gamma-aminobutyric-acid-type-A (GABA-A) receptor is its target. Righting reflex is associated with conscious response. The nucleus basalis (NB) acts as a major relay between the reticular activating system and the frontal cortex (FC). Propofol may mediate righting reflex by affecting GABA-A receptor in NB.

**Methods:**

Fifty male SD rats (250-350 g) were divided into parts I and II. In part I, 20 male SD rats were randomly divided into control group (CG) and NB-lesion group (NG, ibotenic acid-induced NB lesion). In part II, 30 male SD rats were treated with saline (0.9% NaCl, SG group), muscimol (a GABA-A receptor agonist, MG group), and gabazine (a GABA-A receptor antagonist, GG group) in NB, respectively. Two weeks later, the activity of the rats was measured between CG and NG groups. The rats were intravenously injected with propofol (50 mg/kg/h) to test the time of loss of righting reflex (LORR) in all rats. When LORR occurred, the rats received single administration of propofol (12 mg/kg) to measure the time of return of righting reflex (RORR). Electroencephalogram (EEG) activity of the frontal cortex (FC) was recorded.

**Results:**

The numbers of NB neurons were reduced by 44% in the NG group compared to the CG group (*p* < 0.05) whereas the activity of rats was reduced a little in the NG group when compared with the CG group, but the statistical difference was insignificant (*p* < 0.05) whereas the activity of rats was reduced a little in the NG group when compared with the CG group, but the statistical difference was insignificant (*p* < 0.05) whereas the activity of rats was reduced a little in the NG group when compared with the CG group, but the statistical difference was insignificant (*p* < 0.05) whereas the activity of rats was reduced a little in the NG group when compared with the CG group, but the statistical difference was insignificant (*p* < 0.05) whereas the activity of rats was reduced a little in the NG group when compared with the CG group, but the statistical difference was insignificant (*p* < 0.05) whereas the activity of rats was reduced a little in the NG group when compared with the CG group, but the statistical difference was insignificant (

**Conclusions:**

The unilateral NB lesion increased the recovery time and FC delta power, and the NB region might be involved in the emergence after propofol administration. Propofol plays a crucial role for causing conscious loss by affecting GABA-A receptor in NB.

## 1. Introduction

Propofol is a classical intravenous anesthetic and can induce consciousness loss, and the mechanism remains unclear. Basal forebrain (BF) is located in the anterior aspect of the hypothalamus and the ventral medial aspect of the striatum. The anatomical structures include nucleus basalis (NB), substantia innominate (SI), nucleus of the horizontal limb of the diagonal band (HDB), magnocellular preoptic nucleus (MCPO) and medial septum (MS) [1]. The injection of fluorescent protein in BF, which tracks the fiber projection of cholinergic neurons, showed that cholinergic nerve fibers are densely projected to the frontal cortex (FC) [2]; the activation of the neurons can increase the expression of c-fos protein in FC neurons [3]. Cholinergic neurons are mainly distributed in NB, which can accept nerve projections from the hypothalamus and brainstem awakening nerve nucleus while emitting dense projections to the FC^4^. Studies have shown that the acetylcholine content of the cerebral cortex derived from NB is higher than that of the slow-wave sleep in the awake and rapid eye movement sleep, indicating that NB cholinergic neurons play an important role in maintaining wakefulness and regulating sleep-wake cycles [4].

Locus cerulean (LC) acts to maintain and promote wakefulness through NB. Microinjection of norepinephrine into NB resulted in increased muscle strength and involuntary movement with desflurane anesthesia, resulting in transient arousal [4]. Microinjection of histidine in NB reduced the inhibition of ether on cortical EEG in rats while the treatment shortened the anesthesia recovery time [5, 6]. Nonspecific damage to BF resulted in drowsiness and the inhibition of cortical EEG activity, but it did not affect righting behavior in awake state in rats [7]. Recent studies have shown that activation of GABAergic neurons in BF promotes sustained arousal and cortical high-frequency discharge in mice [8]. The NB region contains other types of neurons such as glutamatergic and GABA neurons in addition to cholinergic neurons, but there are few reports of NB regulating general anesthesia awakening, and the mechanism is unclear. We hypothesized that NB participates in the recovery of propofol.

Glutamic-aminobutyric acid (GABA) is a very important inhibitory neurotransmitter found in the central nervous system and can act on two different receptors, GABA-A and GABA-B. The mechanism of activation of the two receptors is different: activation of GABA-A receptor increases the permeability of the cell membrane to chloride, producing inhibitory postsynaptic potential; activation of GABA-B receptor increases K^+^ efflux and decreases Ca^+^ permeability. Activation of GABA-A and GABA-B receptors affects the sleep-wake cycle. Activation of these two receptors reduces slow-wave sleep latency and wake-up time; activation of GABA-A receptors reduces the proportion of fast-eye sleep. This study demonstrated that NB GABA-A receptors played an important role in regulating sleep-wake cycles. Propofol acts mainly on the postsynaptic GABA-A receptor, causing C1-influx and hyperpolarizing the cell membrane, thereby reducing neuronal excitability [9]. Studies have reported that high-dose GABA-A agonists (muscimol, 3 *μ*g/*μ*l) can lead to the disappearance of rat righting behavior; subcutaneous injection of GABA-A receptor antagonist (gabazine) weakens the efficacy of propofol, reducing propofol-induced unconsciousness, and the proportion of rat righting behavior disappeared [10]. However, the role of GABA-A receptors in regulating propofol-wake in NB has not been reported.

An electroencephalograph (EEG) has been used clinically to monitor the depth of anesthesia in patients. As the degree of anesthesia increases, EEG mainly exhibits low-frequency delta waves. Animal experiments also show that in the awake state, the cortex exhibits high-frequency gamma. Slow-wave sleep is characterized by a high-amplitude delta wave, accompanied by a decrease in muscle strength—wave (30-60 HZ). Therefore, EEG recording and microinjection techniques were used to observe the effect of NB microinjection of GABA-A receptor agonist/antagonist on the righting behavior and FC EEG of propofol anesthetized rats and to explore whether GABA-A receptors in the NB region participate in the regulation of propofol.

## 2. Materials and Methods

### 2.1. Reagents

Ibotenic acid (a powerful neurotoxicant and has been used as a potent brain-lesioning agent), muscimol (a GABA-A receptor agonist), and gabazine (a GABA-A receptor antagonist) were purchased from Sigma. Propofol was purchased from AstraZeneca (batch number H20140473). Pentobarbital sodium (it activates GABA-A receptors and enhances GABA-activated currents) was bought from Wuhan Haoyue Pharmaceutical Chemical Co., Ltd. (Wuhan, China).

### 2.2. Animals

This study was carried out in accordance with the principles of the Basel Declaration and the guidelines of the Animal Care and Use Committee of China-Japan Union Hospital of Jilin University. The protocol was approved by the animal research ethics committee of China-Japan Union Hospital of Jilin University. 50 healthy male SPF SD rats, weighing 250-350 g, were purchased from the Medical Laboratory Animal Center of the Third Military Medical University (animal license number: CC2012-0015). The rats were raised in the laboratory SPF animal room and housed in a temperature-controlled room (20 ± 1°C) with a 12 : 12 h light–dark cycle and free access to tap water and food.

### 2.3. Animal Grouping

Fifty healthy male SD rats (250-350 g) were divided into two parts I and II. In part I, twenty male SD rats were randomly divided into the control group (CG, phosphate buffer) and the NB-lesion group (NG, unilateral infusion of 1 *μ*l of 10 *μ*g/*μ*l ibotenic acid in NB). In part II, thirty male SD rats were injected with saline (SG group, 1 *μ*l 0.9% NaCl), muscimol (MG group, 1 *μ*l 0.5 *μ*g/*μ*l) and gabazine (GG group, 1 *μ*l 0.2 *μ*g/*μ*l) in NB.

### 2.4. NB Damage and EEG Electrode Placement

The rats were fixed on a stereotaxic instrument, and after that, anesthesia was injected intraperitoneally with 1% sodium pentobarbital intraperitoneally (50 mg/kg). Using bregma as the reference origin, the coordinates of NB and FC were determined. The NB coordinates (1.4 mm rear, 2.6 mm left, 8.3 mm depth) were placed into the microinjection instrument (0.41 mm OD, 7.8 mm length), FC coordinates (1.4 mm front, 2 mm left, 1.5 mm depth), and the EEG recording electrode was placed. Then, the injection inner tube (the tip is 0.5 mm beyond the outer cannula) connected to the PE tube was placed in the cannula, and the microinjection rate of ibotenic acid was 0.25 *μ*l/min for 4 min. Finally, dental cement was applied to the surface of the skull to fix the EEG recording electrode and the reference electrode. Rats were injected intraperitoneally with penicillin 20 U for three consecutive days to reduce the infection rate. The cage was kept in the SPF animal room of the laboratory.

### 2.5. The Effects NB-Lesion on Motor Activity

After two-week establishment of the NB-lesion model, the behaviors of rats were observed in a series of 10–15 s intervals over the course of a one-hour period of observation between the NG and CG groups. Total motor activity was measured by using a behavioral checklist according to a previous report for independent quantification of movements of the head, mouth, trunk, and limbs [11]. Individual behaviors such as sniffing, licking, biting, gnawing, and vertical posture were scored as present or absent in an interval, and the associated behavioral scores were expressed as the percent of the total number of intervals in which that behavior was observed.

### 2.6. Behavioral and EEG Records

The sequential method was used to determine the ED50 of loss of righting reflex (LORR) induced by propofol. The initial dose of 4 mg/kg was used to start intravenous propofol, and the dose was increased by 1 mg/kg every 30 s until the ratification behavior disappeared. Percentage of rat LORR per dose was calculated according to the formula *Y* = *Y*_min_ + (*Y*_max_ − *Y*_min_)/[1 + 10^log(ED50 − X)∗m^]. The dose-response curve of the disappearance of rat righting behavior was fitted (*Y* represented the percentage of disappearing of the rights behavior, and *X* represented the logarithm of the dose of propofol. ED50 indicated that half of propofol dose when the rats' righting behavior disappeared). LORR was measured by continuous intravenous infusion of propofol (50 mg/kg/h). After LORR occurred, single intravenous administration of propofol (12 mg/kg) and recovery of righting behavior (RORR) transpired. The changes in FC brain electricity under anesthesia with propofol (50 mg/kg/h) were recorded. LORR was defined as placing the rat in the supine position and not change from the supine position to the prone position within 30 s. RORR is defined as the ability to return to normal position within 5 s when the rat is in the supine position, i.e., the four feet are landing at the same time.

Normal EEG is divided into slow-wave sleep delta wave (1-4 HZ) and theta wave (4-8 HZ) according to frequency, alpha wave (8-12 HZ) in awake state, and beta wave (12-25 HZ) in emotional state, and gamma wave (25-60 HZ) in fast-eye movement sleep state. After the propofol was intravenously injected at a dose of 50 mg/kg/h, the EEG was recorded for 20 min. The changes of EEG signals within 15-20 min were compared and analyzed. The electrode in which the FC is placed is the recording electrode, and the electrode in the visual cortex is the reference electrode. The EEG signal was collected by CEDPowerl401, the filtering range (0.1 HZ-0.1 kHZ, gain: 1000x), and Spike2 software processed and analyzed the EEG data.

### 2.7. HE Staining

The sternum of the rat under anesthesia was cut open to fully expose the heart. After perfusion of 0.9% saline 500 ml along the left ventricle, the right heart ear was cut to ensure that the saline flows under the stream. Then, 4 ml of formaldehyde was infused with 300 ml. After the rat tail movement occurred, the flow rate was adjusted to sufficiently fix the tissue. The rat brain tissue was taken out, placed in a 4% formaldehyde solution for 24 h, and then placed in a 30% sucrose solution to sink to the bottom. HE sections of NB (objective 20x) were observed under a microscope, and the number of neurons was counted using Image-Pro Plus 6.0 software.

### 2.8. Evaluation of NB Injury

The preliminary results showed that the eosin dye was microinjected at a rate of 0.25 *μ*l/min, and the total diffusion length of 1 *μ*l was 200 *μ*m. Therefore, one slice was taken at intervals of 40 *μ*m per rat, and a total of 10 brain groups with a thickness of 4 *μ*m were obtained for HE staining. The NB neurons were counted using a circular frame with a radius of 200 *μ*m.

### 2.9. Statistics

The cell count was performed by Image-Pro Plus 6.0 software, and the EEG analysis was performed by Spike2 software. The data were analyzed by SPSS18.0 software, and the graph was drawn by GraphPad Prism6 software. The measurement data were mean values ± standard deviation (S.D.). It was indicated that the independent sample *t* test was used for comparison between groups, and *p* < 0.05 was considered to be statistically significant.

## 3. Results

### 3.1. NB Neuron Damage Effect

H&E stain analysis showed the NB difference between control and IBA-lesion groups (Figures 1(a) and 1(b)). The cell number in the NB region in control (Figure 1(c)) was higher than that in the IBA-lesion group (Figure 1(d)). Compared with the control group, the number of NB cells was reduced by 44% (Figure 1(e), *p* < 0.05), suggesting the injury NB model was successfully established.

After 2-week establishment of the NB-lesion model, no significant differences were observed between NB- and sham-lesioned rats although the total activities in the CG group were slightly lower than those in the NG group (Figure 2(a)). In a similar case, the motor activity was also similar between the two groups during one-hour observation (Figure 2(b)).

### 3.2. Rat Behavioral Determination

Figure 3(a) shows the LORR time determined by continuous pumping of propofol at 50 mg/kg/h.  Figure 3(b) shows the RORR time determined after a single intravenous injection of propofol at 12 mg/kg. The ED50 of propofol-induced LORR was 7.2 ± 0.2 and 7.0 ± 0.4 mg/kg in the CG and NG groups, respectively. The NG reactivity curve was slightly shifted to the left compared to the CG group. However, the difference was insignificant (*p* > 0.05, Figure 3(c)), indicating that NB injury did not affect the sensitivity of propofol. The results showed that compared with the control group, NB injury did not affect the rat LORR time induced by propofol (848 ± 18 s and 859 ± 25 s in the CG and NG groups, respectively, *p* > 0.05, Figure 3(d)). Compared with the CG group, unilateral NB injury significantly prolonged the duration of propofol (718 ± 26 s and 917 ± 31 s in the CG and NG groups, respectively, *p* > 0.05, Figure 3(d)).

### 3.3. FC EEG

In order to determine the optimal dose for propofol, different propofol doses (50, 60, and 70 mg/kg/h) were selected to observe the effects of different doses of propofol on FC EEG in rats.  Figure 4(a) shows that the rat had a high-frequency and low-amplitude alpha wave in awake; 50 mg/kg/h propofol increased the energy of the delta wave (Figure 4(b)); 60 mg/kg/h propofol increased the energy in the 0-10 HZ band while reduced the energy of the gamma wave (Figure 4(c)); 70 mg/kg/h propofol reduced energy in all bands, and EEG exhibited explosive suppression (Figure 4(d)). When the dose of propofol reached 70 mg/kg/h, the respiratory depression was more obvious in rats, and the EEG showed explosive inhibition. Continuous intravenous infusion of 60 mg/kg/h propofol resulted in mild respiratory depression in individual rats. Therefore, 50 mg/kg/h of propofol was selected, rat FC delta wave (0-4 HZ) energy increased, 40-50 HZ band energy slightly reduced, and vital signs were stable.

The propofol was continuously injected intravenously at a dose of 50 mg/kg/h, and the changes in the FC EEG bands were recorded 15-20 min after LORR (Figure 5(a)). Under propofol, the EEG amplitude increased and the frequency slowed in the NG group when compared to that in the CG group, increasing the proportion of the l-4 HZ delta band in the NG group (CG, 0.51 ± 0.04 and NG, 0.75 ± 0.06, *p* < 0.05, Figure 5(b)).

The effect of NB microinjection of saline/muscimol/gabazine on rat FCEEG was also observed under anesthesia with 50 mg/kg/h propofol. NB microinjection was started after 10 min LORR, and propofol was continuously infused to rat for 20 min. Finally, the EEG spectral changes in the 15-20 min period were analyzed. The results showed that rats increased the proportion of 1-4 HZ delta bands in the MG group when compared to that in the SG group (Figure 5(c), SG, 0.51 ± 0.04; MG, 0.70 ± 0.12, *p* < 0.05), reducing the 25-60 HZ gamma band. The ratio in the MG group was higher than that in the SG group (Figure 5(c), SG group: 0.05 ± 0.01; MG group, 0.028 ± 0.02, *p* < 0.05); the rats reduced the energy of the l-4 HZ delta band in the GG group when compared with the SG group (Figure 5(c), SG, 0.51 ± 0.04; GG, 0.35 ± 0.08, *p* < 0.05).

### 3.4. The Effects of NB GABA-A Receptor Behavior in the Rats Anesthetized by Propofol

Figure 6(a) shows that the rat LORR was determined by continuously pumping propofol at 50 mg/kg/h.  Figure 6(b) shows the RORR time of rats after a single intravenous injection of propofol at 12 mg/kg. The ED50 of propofol-induced LORR was 7.2 ± 0.2 mg/kg, 6.9 ± 0.3 mg/kg, and 7.3 ± 0.1 mg/kg in the SG, MG, and GG groups, respectively. Compared to the SG group, the MG group propofol-reactivity curve was slightly left-shifted, and the difference was insignificant (*p* > 0.05, Figure 6(c)); the GG group curve was slightly right-shifted, the difference was insignificant (*p* > 0.05, Figure 6(c)), indicating that the GABA-A receptor in the NB brain region did not affect the sensitivity of propofol.

Saline/muscimol/gabazine treatment did not affect the LORR time (the SG group: 848 ± 18 s, the MG group: 817 ± 54 s, and the GG group, 853 ± 36 s, *p* > 0.05, Figure 6(d)). Compared with the SG group, the gabazine and muscimol significantly prolonged the RORR time (SG, 718 ± 26 s; GG, 519 ± 33 s; MG, 1277 ± 68 s, *p* < 0.05, Figure 6(d)).

### 3.5. The Effects of NB GABA-A Receptor on FC EEG in the Rats Anesthetized by Propofol

Figure 7(a) shows the time of LORR, propofol infusion, and microinjection of saline/muscimol/gabazine in rat NB.  Figure 7(b) shows the original EEG record map. The study also observed the effect of NB microinjection of saline/muscimol/gabazine on rat FCEEG under 50 mg/kg/h propofol.  Figure 7(c) shows the spectrum analysis diagram among the three groups. Compared with the SG group, rats increased the proportion of 1-4 HZ delta band (Figure 7(d), SG, 0.51 ± 0.04; MG, 0.70 ± 0.12, *p* < 0.05), reduced the proportion of 25-60 HZ gamma band in the MG group (SG, 0.05 ± 0.01; MG, 0.028 ± 0.02, *p* < 0.05); rats reduced the energy of the l-4 HZ delta band in the GG group (SG, 0.51 ± 0.04; GG, 0.35 ± 0.08, *p* < 0.05).

## 4. Discussion

Theoretically, NB-lesion will affect motor activity since NB plays an important role in regulating the behavioral state in the neuromodulatory system [12]. However, the present results indicated that NB-lesion caused the loss of some NB cells and affected the motor activity a little after 2-week establishment of the model (Figure 2).

After nonspecific NB injury, prolonged wake-up time and increased FC delta wave in propofol-anesthetized rats indicated that NB was involved in the awakening process. Propofol acts on the GABA-A receptor to exert a sedative and hypnotic effect. Whether propofol exerts its anesthetic efficacy by mediating GABA-A receptors in the NB brain region is less reported. Therefore, we conducted experiments to investigate the activation or antagonism of GABA-A receptors in the NB region and observed the effects of propofol on behavior and cortical EEG. The GABA-A receptor in NB is involved in the regulation of the recovery process and FCEEG activity in propofol-anesthetized rats.

The basal forebrain plays an important role in regulating cortical activity and sleep/awakening: MS cholinergic neurons are densely projected into the hippocampus to regulate the limbic system; NB cholinergic neural crests project to the cortex and amygdala and also project to the thalamic reticular nucleus which indirectly affects cortical activity. Unlike cholinergic neurons, GABAergic neurons that are densely projected into the midbrain dorsal region, dorsal raphe nucleus, and hypothalamus play an important role in regulating sleep and fast-eye-movement sleep. In addition to projecting into the cortex, glutamatergic neurons also form synaptic connections with lateral hypothalamic appetite neurons, maintaining and promoting behavioral arousal (Figure 8) [13]. The NB is a somewhat diffuse collection of large cholinergic and noncholinergic neurons (Figure 8). Cholinergic neurons are the dominant source of acetylcholine to the cerebral cortex, and activate the cortex during both wake and rapid eye movement (REM) sleep status, and play an important role in consciousness, sleep, motor activity, learning, memory, and behavior [14, 15]. Hypnosis is mediated by the changes in hypothalamic-pituitary-adrenal (HPA). The decrease in the HPA activity may reduce stress hypnosis [16]. Noncholinergic neurotransmitters GABA and glutamate play a major role in central integration of HPA stress responses [17]. Glutamate and GABA are quantitatively the most important excitatory and play important roles in sedative and hypnotic activities [18].

Studies have shown that cholinergic neurons play an important role in regulating cortical activity and sleep/wake. The 192 IgG-saporin-specific NB injury cholinergic neurons increase the recovery behavior of rats with propofol and pentobarbital. However, it did not affect the induction time of anesthesia [19]. NB microinjection of orexin A cannot only increase the content of cortical acetylcholine but also reduce the inhibitory effect of isoflurane on cortical EEG and shorten the recovery time of propofol [20]. Interestingly, after specific NB injury of cholinergic neurons, microinjection of orexin A was sufficient to maintain arousal in rats [21]. This also indicates that noncholinergic neurons of NB also play an important role in regulating sleep-wake states.

Therefore, we used IBA nonspecific damage to unilateral NB to observe the effect of propofol induction/wake time and FC brain electricity. The present results showed that NB injury prolonged the recovery time of propofol treatment and increased the proportion of FCl-4 HZ delta band. We hypothesized that the regulation of the ventral reticular activation system after NB injury was impaired, which weakened the nerve projection of NB to a certain extent, and thus reduced the activity of FC neurons, i.e., the increase in the proportion of low-frequency high-delta band. The damage to the ventral tegmental dopaminergic neurons significantly increased propofol recovery time but did not change propofol sensitivity and induction time [22]. Just like our results, the sensitivity and induction time of propofol were not affected after NB injury, indicating that anesthesia recovery is not a reverse process of anesthesia induction. Therefore, NB is involved in the regulation of the awakening process after propofol treatment.

Local neuronal activation can be achieved by microinjection of specific chemical drugs or electrical stimulation. For example, GABA-A receptor antagonist (gabazine) can alleviate the inhibition of general anesthetics, thereby exciting the degree of neuronal neuron excitation. Depending on the diffusion range of the drug, according to the results of the first part, the microinjection speed of the experimental drug was set at 0.25 *μ*l/min, the total amount was l *μ*l, and the diffusion radius was 213 ± 8 *μ*m.

The main target of propofol is the GABA-A receptor. Nelson et al.' studies have shown that microinjection of muscimol into the nodular papillary nucleus can cause dose-dependent sedation in rats, and gabazine increases propofol-treated recovery time, while LC and thalamus did not produce significant effects, suggesting that the nodular papillary nucleus plays a key role in the regulation of propofol [10]. Microinjection of histidine in NB increased the proportion of arousal time and caused cortical electrical arousal. These data suggest that NB is an important site for histidine to promote cortical arousal [23]. However, whether the GABA-A receptor in the NB brain region is involved in the regulation of propofol-awakening has not been reported yet.

GABAergic neurons in the BF brain region are subdivided into parvalbumin+ (*p*V+) GABAergic neurons and somatostatin+ (SOM+) GABAergic neurons [13]. Min uses optogenetic studies which showed that the synapses were interrelated between neurons in the BF brain: glutamatergic neurons, PV+GABAergic neurons, and cholinergic neurons emit excitatory projections to SOM+GABA neurons; SOM+GABAergic neurons emit inhibitory projections to cholinergic neurons and glutamatergic neurons; cholinergic neurons and PV+GABAergic neurons simultaneously receive excitatory projections of glutamatergic neurons. The above studies have described the interactions between different types of neurons in BF, and this study used electrophysiological techniques to investigate whether propofol regulates rat behavior and prefrontal EEG via NBGABA-A receptors.

The present results showed that NB microinjection of muscimol prolonged the awakening time of propofol and decreased the excitability of FC neurons, mainly due to the increase of delta wave proportion and the decrease of the proportion of gamma wave. We hypothesized that muscimol acted on GABA-A receptors in cholinergic, glutamatergic, and PV+GABAergic neurons reduced the activity of awakening neurons and enhanced the efficacy of propofol. NB microinjection of gabazine accelerated the awakening time of propofol and increased the excitability of FC, mainly due to the decrease of delta wave proportion. However, gabazine blocked the inhibitory effect of propofol on the awakening neurons by acting on the GABA-A receptors in cholinergic, glutamatergic, and PV+GABAergic neurons.

There was some limitation in the present work: the nonspecific NB injury neurons in this study did not clarify the role of specific neurons in propofol; only the GABA-A receptor was investigated in NB and other types of receptors were not explored in NB. A more specific approach, such as Designer Receptors Exclusively Activated by Designer Drugs (DREADDs), will be used to study the mechanism, by which specific neurons in NB regulate the time of awakening after propofol treatment.

## 5. Conclusion

Nonspecific NB injury prolonged the awakening time of propofol treatment and increased the proportion of FC delta wave, indicating that NB participated in the awakening process of propofol treatment. NB microinjection of GABA-A receptor agonist (muscimol) inhibited FC brain electrical activity and prolonged the awakening time of propofol; GABA-A receptor antagonist (gabazine) increased FC brain electrical activity and shortened propofol recovery time. It suggested that GABA-A receptors in NB are involved in the regulation of the recovery of consciousness in propofol-anesthetized rats.

## Figures and Tables

**Figure 1:** H&E stain analysis of NB between control and IBA-lesion groups: (a) control group, (b) IBA-lesion group, (c) the cell in the NB region in the control group, and (d) the cell in the NB region in the IBA-lesion group. (e) The comparison of NB cell number between control and IBA-lesion groups. 3 V, three ventricle; O, supra optic nucleus. Compared with the control group, *p* < 0.05 and there was a significant difference.

**Figure 2:** Behaviors induced by lower doses of ibotenic acid in sham- and nucleus basalis-lesioned rats (*n* = 10, each case). (a) % of intervals in which behavior observed. (b) Proportion of animals expressing motor activity in consecutive 15 s observation intervals within one hour.

**Figure 3:** Effect of NB on propofol dose-response curve and rat LORR/RORR time. Note: (a) Schematic diagram of LORR in rats by continuous intravenous pumping of propofol (50 mg/kg/h). (b) Schematic diagram of RORR in rats by single intravenous injection of propofol. (c). The LORR reactivity curve of the rats in the destructive group caused by propofol slightly shifted to the left, but the difference was not statistically significant. (d) Effect of NB on rat LORR and RORR time. *p* < 0.05, and there was a significant difference compared to the control group.

**Figure 4:** EEG and energy spectrum analysis of prefrontal cortex in rats with different anesthetic doses of propofol. (a) Record of the high-frequency low-level alpha wave in the awake state and the energy spectrum in the right. (b) Low doses of propofol (50 mg/kg/h) increase the slow wave energy as an increase in delta wave energy, expressed in black. (c) indicates that a medium dose of propofol (60 mg/kg/h) increases the energy in the 0-10 Hz band, reducing the energy of the 50-60 HZ fast wave, producing a mild inhibition, indicated in black. (d) indicates a dose of 70 mg/kg/h.

**Figure 5:** Comparison of EEG recordings in the prefrontal cortex of rats. The control of IBO-lesion groups. Under anesthesia with 50 mg/kg/h propofol, EEG of (a) the normal group and (b) the damaged group. (c) The increase of the 0-10 Hz band of the damaged group. (d) The statistical diagram of the energy of each frequency band; the delta wave proportion of the damaged group increases. There was a significant difference compared to the CG group if *p* < 0.05.

**Figure 6:** Rat NB microinjection of saline/muscimol/gabazine, propofol dose-response curve, and rat LORR/RORR time changes. (a) Schematic diagram of rat LORR was determined by continuous injection of 50 mg/kg/h propofol. (b) RORR was determined by intravenous injection of 12 mg/kg propofol. (c) After NB microinjection of the drug, the dose-response curve of propofol was determined. (d) Chart of LORR/RORR time. *p* < 0.05 compared with the saline group, and there was a significant difference.

**Figure 7:** Changes in prefrontal cortex EEG after rat NB microinjection of saline/muscimol/gabazine. (a) EEG recording schematic. (b) EEG original record map. (c) Spectrum analysis of diagram among the three groups. (d) Statistical chart of each frequency band of EEG. ^∗^*p* < 0.05 compared to the saline group, and there was a significant difference.

**Figure 8:** Neuroprojection of the nucleus basalis (NB). The NB of the basal forebrain plays an essential role for regulating behavioral state in the neuromodulatory system. Red and blue markers indicate cholinergic and noncholinergic neurons, respectively.

## Data Availability

The data for the current study are available from the corresponding author upon reasonable request.
